This article has been retracted.

# miR-451a Inhibited Cell Proliferation and Enhanced Tamoxifen Sensitive in Breast Cancer via Macrophage Migration Inhibitory Factor

**DOI:** 10.1155/2015/207684

**Published:** 2015-06-16

**Authors:** Zhenru Liu, Tianyu Miao, Ting Feng, Zhouhua Jiang, Mingyuan Li, Liming Zhou, Hong Li

**Affiliations:** ^1^Key Laboratory of Obstetric & Gynecologic and Pediatric Diseases and Birth Defects of Ministry of Education, West China Second University Hospital, Sichuan University, Chengdu 610041, China; ^2^Department of Pharmacology, West China School of Preclinical and Forensic Medicine, Sichuan University, Chengdu, Sichuan 610041, China; ^3^West China School of Medicine, Sichuan University, Chengdu 610041, China; ^4^985 Science and Technology Platform for Innovative Drugs of Sichuan University, Chengdu 610041, China

## Abstract

This study aims to investigate the regulative effects of microRNA-451a (miR-451a) on cell proliferation and sensitivity to tamoxifen in breast cancer cells. In cell culture experiments, the lentiviral vectors of pHBLV-miR-451a and pHBLV-miR-451a sponge were constructed and used to transfect MCF-7 and LCC2 cells. The transfection efficiency was tested by fluorescent observation, and cell lines with stable over- or downregulated expression of miR-451a were established. The expression of miR-451a and the target gene macrophage migration inhibitory factor (MIF) were detected by real-time reverse transcriptase polymerase chain reaction and/or western blot. Moreover, MTT assay, colony formation, and Transwell invasion assays were also performed. Data showed that the recombinant lentiviral vectors were constructed correctly, and the virus titer was 1 × 10^8^ CFU/mL. The stable transfected cells were obtained. Overexpression of miR-451a downregulated MIF expression in mRNA and protein levels and inhibited cell proliferation, colony formation, and invasion of breast cancer cells. Downregulation of miR-451a upregulated MIF expression and increased breast cancer cell growth, invasion, and tamoxifen sensitivity. In summary, the miR-451a/MIF pathway may play important roles in the biological properties of breast cancer cells and may be a potential therapeutic target for breast cancer.

## 1. Introduction

MicroRNAs (miRNAs) are noncoding small RNAs (19–25 ribonucleotides) that can regulate gene expression at transcriptional and posttranscriptional levels by binding to the 3′-untranslated regions (3′UTRs) of target mRNA [1]. miRNAs have been reported to be involved in a range of biological processes, including cell proliferation and apoptosis. Altered miRNAs expressions were likely to contribute to human diseases including cancers [2]. To date more than 900 miRNAs have been identified, but the functions and mechanisms of many of them in cancers remain to be determined [3]. miR-451a is located on chromosome 17q11.2, a region that is amplified in some types of carcinomas [4]. Previous studies have demonstrated that miR-451a inhibited cell growth and proliferation and enhanced the activity of anticancer drugs [5, 6].

Macrophage migration inhibitory factor (MIF) is a proinflammatory cytokine that is involved in carcinogenic transformation and cancer development. The MIF levels are increased in a number of cancers including breast cancer and contribute to the survival and homeostasis control of cancer cells [7].

Breast carcinoma is the most frequent malignant neoplasm diagnosed in women, and approximately 70% of this cancer expresses the estrogen receptor (ER). Tamoxifen is the most common and effective treatment for patients with ER*α*-positive breast cancers, which significantly reduces disease progression and is associated with preferable impact on survival of patients [8]. However, almost 50% of patients with advanced breast cancer do not respond to tamoxifen treatment. Furthermore, a lot of patients treated with tamoxifen suffer relapses, even when the initial responses are positive [9, 10]. It has been reported that altered expression of specific miRNAs is responsible for tamoxifen resistance, which can be used to predict the outcomes and responses to treatment in breast cancer patients [11]. Furthermore, the acquisition of tamoxifen resistance in breast cancer cells was accompanied by a significant increase in the cells' invasive ability. In order to explore the functions of miR-451a in breast cancer cells, we established recombinant lentiviral vectors with over- or downexpression of miR-451a, and the vectors were used to transfect MCF-7 and LCC2 breast cancer cells. Functional studies showed that miR-451a downregulated MIF expression, inhibited cell proliferation and invasion, and increased tamoxifen sensitivity of these breast cancer cells.

## 2. Materials and Methods

### 2.1. Construction of Transfer Vectors pHBLV-miR-451a and pHBLV-miR-451a Sponge

We used the lentiviral vectors of pHBLV, pSPAX2, and pMD2G, which were a transfer vector, packaging plasmid, and envelope plasmid, respectively. For lentivirus construction, the sequence of mature miR-451a (5′-AAACCGUUACCAUUAC-UGAGUU-3′) was obtained from miR-Base (http://www.mirbase.org/). The pre-miR-451a and miR-451a sponge oligonucleotides were chemically synthesized by Sunny Biotech Co., Ltd., Shanghai, China, and the primers were as follows: pre-miR-451a F: 5′-ACAGGATCCCTGGAGCCTGACAAGG-3′ (EcoRI restriction site is underlined points), pre-miR-451a R: 5′-ATTGAATTCAAAAAAGCCCCCA-CCCCTGCCTT-3′ (BamHI restriction site is underlined points), miR-451a sponge F: ACAGGATCCAACTCAGTAATGGTAACGGTTTGCTAGAACTCAGTAATGG-TAACGGTTTGCTAGAACTCAGTA, and miR-451a sponge R: ATCGAATTCAAACC-GTTACCATTACTGAGTTCTAGCAAACCGTTACCATTACTGAGTTCTAGCAAA-CCGTT. Then the recovered PCR products with precursor sequence for miR-451a self-complementary miR-451a sponge were inserted into pHBLV-U6-ZsGreen-Puro lentiviral vectors (Hanbio, Shanghai, China). After the pre-miR-451a and miR-451a sponge lentiviral-based vectors were transformed to DH5*α* cells, antibiotic-resistant colonies were selected on LB-ampicillin agar plates. The plasmid containing the target gene was verified by PCR, double digestion, and DNA sequencing.

### 2.2. Cell Lines and Culture

Human embryonic kidney- (HEK-) 293T cells and human breast cancer cell lines (MCF-7 and LCC2 cells) were obtained from Shanghai Institute of Cell Biology (CAS, China) and cultured in DMEM medium supplemented with 10% fetal bovine serum (FBS, HyClone, Logan, UT), 100 kU/L^−1^ penicillin, and 100 mg/L^−1^ streptomycin at 37°C in a humidified incubator with 5% CO_2_. The tamoxifen-resistant cells LCC2 were cultured in the presence of 10^−12^ M 4-hydroxytamoxifen (4-OHT, Sigma-Aldrich, St. Louis, MO, USA) to maintain the resistant properties.

### 2.3. Packaging and Purification of Lentiviral Particles

The logarithmic of HEK-293T cells were trypsinized, and the cell density was adjusted to 1.5 × 10^6^ cells/mL with complete medium. The cells were reseeded into T75 cell culture flasks and cultured for 24 h. The cells were 80%–90% confluent on the day of transfection. The recombinant vectors encoding miR-451a or miR-451a sponge and packaging plasmids (pSPAX2 and pMD2G) were cotransfected into HEK-293T cells with LipoFiter (Hanbio, Shanghai, China). After 6 h transfection, the cell culture medium was replaced by fresh complete DMEM. The expression of ZsGreen was determined after 24 h transfection, and the culture supernatant was collected after 48 h transfection and centrifuged at 4,000 ×g for 10 min to remove any cell debris sedimentation. Then the supernatant was filtered through a 0.22 *μ*m cellulose acetate filter and centrifuged at 72,000 ×g for 120 min at 4°C to harvest the high-titer lentivirus containing miR-451a or miR-451a sponge gene. The lentivirus without transgene was produced in the same way and used as negative control.

### 2.4. Determination of Virus Titer

The HEK-293T cells were seeded into 96-well plates at 1.0 × 10^3^ cells per well. After 24 h, the media were replaced with serial diluted virus solution, and the cells were cultivated under the conditions of 5% CO_2_ and 37°C. After 72 h, the number of fluorescent cells and total cells were counted under microscope. The titer of virus was acquired using the appropriate dilution.

### 2.5. Virus Transfection and Selection of Stable Transfected Cell Line

Logarithmic phases of MCF-7 and LCC2 cells were cultured at 1 × 10^5^ cells per well in 24-well plates and divided into blank control, Lv-negative control Lv-miR-451a, and Lv-miR-451a sponge. After 24 h, the mixture of appropriate volume of virus stock solution and cell culture medium was added to cells. After 24 h incubation, the virus solution was removed and replaced with complete medium. To establish stable transfected cell lines, 72 h after transduction, puromycin was added to the medium at the concentration of 5 *μ*g/mL. After antibiotic selection for 3 weeks, the blank control cells were completely dead, and the corresponding stable transfected cell lines were obtained.

### 2.6. Detection of miR-451a and MIF Gene Expression by Real-Time RT-PCR

Total RNAs from MCF-7 and LCC2 Cells were prepared using the Trizol reagent (Invitrogen, Carlsbad, CA) after the viral transduction. RevertAid First Strand cDNA Synthesis Kit (Fermentas, Burlington, ON, Canada) was used for the reverse transcription of total RNA (0.1 *μ*g) according to the manufacturer's instructions. Real-time PCR was performed using the SYBR Green Master Mix (Takara Bio Inc.). Primers were used as follows: miR-451a (F: 5′-ACACTCCAGCTGGGAA-ACCGTTACCATTACT-3′; R: 5′-CTGGTGTCGTGG AGTCGGCAA-3′), U6 (F: 5′-CTCGCTTCGGCAGCACA-3′; R: 5′-AACGCTTCACGAATTTGCGT-3′), MIF (F: 5′-GCAGAACCGCTCCTACAGCA-3′; R: 5′-GGCTCT-TAGGCGAAGGTGGA-3′), and *β*-actin (F: 5-′CCTGGCACCCAGCACAAT-3′; R: 5′-GGGCCGGACTCGTCATACT-3′). All the reactions were performed in triplicate using the ABI Prism 7500 real-time PCR system (Applied Biosystem, Foster City, CA, USA). The data were expressed as 2^−ΔΔCt^.

### 2.7. Cell Proliferation Assay

Cell proliferation was measured by MTT assay. MCF-7 and LCC2 cells transfected with scrambled oligonucleotide, miR-451a, or miR-451a sponge were seeded into 96-well plates (6 × 10^3^ cells/well) and treated with 4-OHT at different concentrations for 48 h. 20 *μ*L MTT (5 mg/mL) was added into each well and incubated for 4 h. After the media were removed, 150 *μ*L DMSO (Sigma-Aldrich, St. Louis, MO, USA) was added to each well to dissolve the formazan crystal. The absorbance was measured at 490 nm with a microplate reader (Bio-Rad, Hercules CA). The concentration of 4-OHT yielding 50% growth inhibition (IC_50_) was calculated using medium effect algorithm with three independent experiments [12].

To draw the cell growth curve, MCF-7 and LCC2 cells were seeded into 96-well plates (3 × 10^3^ cells/well); after transfection, MTT assay was performed to detect cell survival at Days 1, 2, 3, 4, 5, 6, and 7, and optical density (OD) was measured at 490 nm.

### 2.8. Colony Formation Assay

MCF-7 and LCC2 cells were plated at a low density (5 × 10^3^ cells per 10 cm plate) after transfection and incubated for 14 days at 37°C and 5% CO_2_ in a humidified atmosphere. Colonies were fixed with 90% ethanol, stained with crystal violet, and counted under inverted microscope.

### 2.9. Transwell Invasive and Wound Healing Assay

Transwell chambers (Corning) with 8 *μ*m pore size were coated with Matrigel (BD Bioscience) on the upper surface. 200 *μ*L MCF-7 and LCC2 cells suspension with the recombinant lentiviral vector was plated into the upper chambers, and the medium with 10% FBS was piped into the lower Transwell chamber. After 24 h, the cells that had invaded through the membrane to the lower chambers were fixed with 90% ethanol and stained and counted under inverted microscope (400x).

Cells were seeded into 6-well plate about 24 h. When the cells grew to over 90% confluence, they were wounded by scratching with a pipette tip and washed with PBS for three times. Cells were refreshed with 2.5% FBS and photographed after 24 h and 48 h incubation at 37°C.

### 2.10. Western Blot

Cells transfected with lentiviral vectors were lysed with lysis buffer at 4°C for 30 min. The protein concentration was measured by the Bio-Rad assay system (Bio-Rad Hercules, CA, USA). The same amount of proteins (50 *μ*g) was separated on 9% SDS-PAGE and transferred to PVDF membrane (Bio-Rad Hercules, CA, USA). The membrane was blocked by 5% nonfat milk at room temperature for 1.5 h, incubated with rabbit monoclonal anti-MIF antibody (1 : 1000, Abcam) at 4°C overnight, and then washed with PBST followed by incubation with the second antibody (goat anti-rabbit IgG, 1 : 2000, Boster, Wuhan, China) at room temperature for 1.5 h. The signal was detected using Chemiluminescence Kit (Millipore Corporation, Billerica, MA, USA). The intensity of the bands was quantitated using the Image Gel Documentation System, and data were presented as the relative pixel density normalized to GAPDH [13].

### 2.11. Statistical Analysis

The data were presented as mean ± SD. Experimental data were analyzed by one-way analysis of variance (ANOVA), and statistical analysis was performed with SPSS 16.0 software. Significance was defined by *P* < 0.05.

## 3. Results

### 3.1. PCR Amplification and Sequencing of Pre-miR-451a and miR-451a Sponge Fragments

DNA fragments of pre-miR-451a and miR-451a sponge were successfully amplified by PCR. Electrophoresis showed the specific bands of pre-miR-451a and miR-451a at 243 bp and 88 bp, respectively (Figures 1(a) and 1(b)). The sequences of pre-miR-451a and miR-451a sponge were also analyzed (Figures 1(c) and 1(d)).

### 3.2. Lentivirus Packaging and Transduction of MCF-7 and LCC2 Cells

HEK-293T cells were cotransfected with the transfer plasmid, pHBLV-transgenes, the envelope plasmid (pMD2G), and the packaging plasmids (pSPAX2). The virus titer was calculated by the formula virus titer = 3 × 10^4^ × 12% × 30 × 10^3^ = 1.08 × 10^8^ PFU/mL. ZsGreen was expressed after MCF-7 and LCC2 cells were transduced with the lentivirus. After selection for 3 weeks by puromycin, we obtained stable transfected cell lines of MCF-7 and LCC2 cells. All the MCF-7 cells with ZsGreen expression were observed under microscope (Figure 2), and LCC2 cells were also observed (data not shown).

### 3.3. The Expression of miR-451a and MIF before and after Transfection in MCF-7 and LCC2 Cells

We performed real-time RT-PCR to test the expression of miR-451a and MIF. The expression of miR-451a was significantly lower, but the mRNA expression of MIF was significantly higher in LCC2 cells compared with MCF-7 cells (Figure 3(a)). After cell transfection, the expression of miR-451a was significantly increased in Lv-miR-451a group, whereas it significantly decreased in Lv-miR-451a sponge group compared with the Lv-miR-451a NC (*P* < 0.05) in both of MCF-7 and LCC2 cells (Figure 3(b)). Thus, we established the stable transfected cell lines of MCF-7-miR-451a, MCF-7-miR-451a sponge, LCC2-miR-451a, and LCC2-miR-451a sponge. Furthermore, overexpression of miR-451a significantly decreased the MIF mRNA expression. In contrast, downregulation of miR-451a significantly increased MIF mRNA expression (Figure 3).

### 3.4. miR-451a Suppressed MCF-7 and LCC2 Cell Proliferation and Colony Formation

MTT assay showed that the cell proliferation of MCF-7 (Figure 4(a)) and LCC2 cells (Figure 4(b)) transfected with Lv-miR-451a was significantly decreased compared with negative control (NC). Colony formation assay showed that the proliferation and colony numbers of the cells transfected with Lv-miR-451a were significantly decreased compared to negative control (NC) (Figure 4(c)). In contrast, the proliferation and colony formation were significantly increased in MCF-7 and LCC2 cells transfected with Lv-miR-451a sponge compared with Lv-miR-451a NC.

### 3.5. miR-451a Suppressed the Invasion Ability of MCF-7 and LCC2 Cells

We first compared the invasion ability of MCF-7 and LCC2 cells at baseline and found that LCC2 cells were more aggressive than MCF-7 (Figure 5(a)). Next we measured the invasion ability of the cells after transfection with Lv-miR-451a, Lv-miR-451a sponge, or Lv-miR-451a NC. The results showed that transfection with Lv-miR-451a significantly inhibited the invasive ability in both of MCF-7 and LCC2 cells compared to Lv-miR-451a NC transfected cells (Figure 5(b)). On the other hand, the invasion ability of the cells transfected with Lv-miR-451a sponge was significantly enhanced compared with those transfected with Lv-miR-451a NC (Figure 5(b)).

### 3.6. Ectopic Expression of miR-451a Partially Increased the 4-OHT Sensitivity of MCF-7 and LCC2 Cells

To understand whether the transfected cells have different responses to 4-OHT, the cells were treated with different concentrations of 4-OHT and cell survival rate was measured. The inhibition rate of cellular survival was significantly increased and the IC_50_ value significantly decreased in both of MCF-7 and LCC2 cells transfected with Lv-miR-451a compared to Lv-miR-451a NC transfected cells. However, the inhibition rate of cellular survival was much lower and IC_50_ was higher in cells transfected with Lv-miR-451a sponge compared with those transfected with Lv-miR-451a NC (Figure 6). All these results confirmed that cells transfected with Lv-miR-451a would restore their sensitivity to 4-OHT, whereas the cells transfected with Lv-miR-451a sponge acquired the drug resistance.

### 3.7. Ectopic Expression of miR-451a Regulated MIF Expression in MCF-7 and LCC2 Cells

Western blot was used to detect MIF expression, and the results showed that MIF protein level was significantly decreased in both MCF-7 and LCC2 cells transfected with Lv-miR-451a and significantly increased in cells transfected with Lv-miR-451a sponge compared with Lv-miR-451a NC and control group. There was no significant difference between Lv-miR-451a NC and control groups (*P* > 0.05) (Figure 7).

### 3.8. MIF Regulated the Cells Invasion and Tamoxifen Sensitivity of LCC2 Cells

In order to determine whether MIF could regulate the breast cancer cells invasion and tamoxifen sensitivity, we transfected LCC2 cells with siMIF and siNC (negative control) and found that siMIF significantly reduced the cell invasion and motility. MTT assay results also showed that siMIF significantly increased the cell survival inhibition rate of 4-OHT, consequently decreased the IC_50_ value, and partially restored the tamoxifen sensitivity of LCC2 cells (Figure 8).

## 4. Discussion

Gene transfection is a process in which nucleic acids are transported into cells and maintain their biological functions in the cells. At present, plasmid vectors and virus vectors are widely used as gene carriers in various studies to explore the roles of miRNAs in the regulation of gene expression, signal transduction, and gene therapy research. Lentiviral vector is designed based on the transformation of HIV-1 production and can be used for both dividing and nondividing cells with the advantages of integrating large exogenous gene into the host chromosome, stable expression, small immune response, and safety [14]. In this study, we established lentiviral expression vectors of Lv-miR-451a and Lv-miR-451a sponge and therefore built a foundation for efficient and stable transfection of MCF-7 and LCC2 cells.

Recently, miRNAs have been demonstrated to play important roles in maintaining normal cellular functions, and the dysregulation of miRNAs could lead to the initiation and progression of tumors [15, 16]. miR-451 (also named as miR-451a) was downregulated in several tumors, such as breast cancer, lung cancer, and gastric cancer [5, 17, 18]. Furthermore, the abnormal expression of miR-451a was involved in the functions of cancer cells, including cell proliferation and survival, migration, and invasion [17, 18]. Each miRNA has hundreds of target genes and has the ability to harbor the target sequence in their 3′-untranslated region (UTR) segment to the seed region of the miRNA [1]. Several targets of miR-451a have been identified, and MIF was verified as one of them using luciferase reporter gene assay in previous study [18]. A number of studies showed that MIF expression was upregulated in various tumors, which can promote cell proliferation and invasion and correlate with worse survival prognosis [19]. However, only a few reports have been presented regarding the MIF function in breast cancer. In order to have a better understanding of the function of miR-451a/MIF pathway in breast cancer, in this study we first detected the miR-451a and MIF expression in MCF-7 and LCC2 cells. We found that miR-451a was decreased but MIF was increased in LCC2 cells compared to MCF-7, which were negative correlation, and LCC2 cells were more aggressive than MCF-7. We next established and verified the stable over- or downregulated expression of miR-451a by transducing Lv-miR-451a or Lv-miR-451a sponge into MCF-7 and LCC2 cell lines. Consequentially, up- or downregulation of miR-451a decreased or increased MIF mRNA and protein expression in these cells, respectively. Furthermore, we found that the cell proliferation and colony formation were suppressed by miR-451a upregulation but increased by miR-451a downregulation. Moreover, miR-451a overexpression inhibited the cell invasive capacity, and the opposite results were found in the cells with downexpression of miR-451a. Our findings are consistent with previous studies in nasopharyngeal carcinoma [20]. Several studies also indicated that MIF was indirectly involved in promoting cancer growth and progression, while depleting endogenous MIF caused a >40% reduction in cancer cell growth in colon cancer [21–23].

The use of most of the anticancer drugs, including tamoxifen, is limited due to the drug resistance by breast cancer cells, which is a serious problem in treating breast cancer patients with positive ER*α* expression, as evidences showed that the expression of estrogen receptor (ER*α*) determined the response of breast cancer cells to tamoxifen [24–26]. The relation between MIF expression level and ER/PR status has been reported, which indicated that JAB1 was a binding partner of MIF and interacted with ER and PR [27]. The altered expression of miRNAs was involved in tamoxifen resistance development and predicted the therapeutic response in breast cancer patients [11]. Previous studies suggested that downregulation of miR-451a might be the mechanism of developing resistance to tamoxifen therapy [5]. Our study showed that miR-451a overexpression in MCF-7 and LCC2 cells enhanced the cell survival inhibition rate and restored the sensitivity to tamoxifen to some extent based on the changes of IC_50_ value. miR-451a may play an important role in chemotherapy resistance as well, and upregulation of miR-451a enhanced the cisplatin and doxorubicin effectiveness [28]. In addition, our study indicated that miR-451a could negatively regulate the MIF protein expression, which is consistent with the finding in gastric cancer [18]. These results suggested that upregulation of MIF induced by downregulation of miR-451a may be one of the underlying mechanisms of tamoxifen resistance in breast cancer. In this study, we used siRNA to study MIF function according to previous studies [29] and found that siMIF significantly reduced the cell invasion and motility, also decreased the IC_50_ value, and partially restored the tamoxifen sensitivity of LCC2 cells. In this sense, our study demonstrated that the inverse correlation between miR-451a and MIF might play important roles in breast cancer. This is the first report to show that miR-451a can suppress cell invasive ability and enhance tamoxifen sensitivity in breast cancer cells.

In summary, in the current study we constructed the lentiviral vectors of miR-451a and established stable transfected cell lines. The functional studies indicated that miR-451a, as a tumor suppressor, had important functions in breast cancer progression through MIF pathway. Further in vitro and in vivo studies are warranted to explore the molecular mechanisms of miR-451a/MIF pathway in breast cancer.

## Figures and Tables

**Figure 1:** Electrophoresis of PCR products and sequencing analysis of pre-miR-451a and miR-451a sponge. (a) and (b) Electrophoresis indicated the specific bands of pre-miR-451a and miR-451a at 243 bp and 88 bp; (c) and (d) sequencing results indicated that the pre-miR-451a and miR-451a sponge sequences were correct.

**Figure 2:** MCF-7 cells transduced by lentivirus after puromycin selection (×200). (a), (c), and (e) Light microscopy of Lv-miR-451a NC, Lv-miR-451a, and Lv-miR-451a sponge; (b), (d), and (f) fluorescent microscopy of Lv-miR-451a NC, Lv-miR-451a, and Lv-miR-451a sponge. All the cells with ZsGreen expression and the stable cell lines were obtained (note: NC means negative control; Lv means lentivirus).

**Figure 3:** The expressions of miR-451a and MIF were examined by real-time PCR. (a) total RNA extracted from the cell lines of MCF-7 and LCC2 was subjected to real-time PCR with miR-451a-specific or MIF-specific primers. The miR-451a expression or MIF mRNA expression was normalized to U6 or GAPDH expression. ^*∗*^ *P* < 0.05 versus MCF-7 cell; (b) total RNA extracted from the stable cell lines of MCF-7 and LCC2 was subjected to real-time PCR with miR-451a-specific primers. The induction of miR-451a expression was normalized to U6 expression; (c) total RNA extracted from these cells was subjected to real-time PCR with MIF-specific primers. The induction of MIF mRNA expression was normalized to GAPDH expression. ^*∗*^ *P* < 0.05 versus Lv-miR-451a NC (MCF-7); ^#^ *P* < 0.05 versus Lv-miR-451a NC (LCC2) (note: NC means negative control; Lv means lentivirus).

**Figure 4:** Effect of miR-451a and miR-451a sponge on cell proliferation and colony formation of MCF-7 and LCC2 cells. Cell proliferation was examined by MTT assay for MCF-7 cells (a) and LCC2 cells (b) transfected with Lv-miR-451a, Lv-miR-451a sponge, or Lv-miR-451a NC. (c) Colony formation was examined for MCF-7 cells and LCC2 cells transfected with Lv-miR-451a, Lv-miR-451a sponge, or Lv-miR-451a NC. ^*∗*^ *P* < 0.05 versus Lv-miR-451a NC (MCF-7); ^#^ *P* < 0.05 versus Lv-miR-451a NC (LCC2) (note: NC means negative control; Lv means lentivirus).

**Figure 5:** Effects of miR-451a and miR-451a sponge on cell invasion ability. (a) The invasion ability of MCF-7 and LCC2 cells. ^*∗*^ *P* < 0.05 versus MCF-7 cell; (b) representative images of the invasion of MCF-7 and LCC2 cells transfected with Lv-miR-451a sponge or Lv-miR-451a. ^*∗*^ *P* < 0.05 versus Lv-miR-451a NC (MCF-7); ^#^ *P* < 0.05 versus Lv-miR-451a NC (LCC2) (note: NC means negative control; Lv means lentivirus).

**Figure 6:** Effects of miR-451a and miR-451a sponge on cell survival and 4-OHT sensitivity in breast cancer cells. (a-b) MTT assay was performed to test cell survival inhibition rate in MCF-7 (a) and LCC2 (b) cells after being transfected with Lv-miR-451a or Lv-miR-451a sponge or Lv-miR-451a NC and treated with different concentrations of 4-OHT; (c) IC_50_ value of 4-OHT was determined after cells were transfected with Lv-miR-451a or Lv-miR-451a sponge or Lv-miR-451a NC. ^*∗*^ *P* < 0.05 versus Lv-miR-451a NC (MCF-7); ^#^ *P* < 0.05 versus Lv-miR-451a NC (LCC2) (note: NC means negative control; Lv means lentivirus).

**Figure 7:** Expression of MIF in each group. The MCF-7 and LCC2 cells were transfected with Lv-miR-451a or Lv-miR-451a sponge or Lv-miR-451a NC. Total lysates were prepared and subjected to western blot with anti-MIF antibody. ^#^ *P* < 0.05 versus Lv-miR-451a NC or control (MCF-7); ^*∗*^ *P* < 0.05 versus Lv-miR-451a NC or control (LCC2) (note: NC means negative control; Lv means lentivirus).

**Figure 8:** MIF was involved in breast cancer cells invasion and tamoxifen sensitivity. (a) After wounding cells were cultured for another 24 h or 48 h, siMIF increased the area of unhealed cell wound size; (b) LCC2 cells were seeded into a Matrigel-coated membrane and cultured for 24 h; siMIF reduced the number of invading cells compared to the siNC; (c) MTT assay indicated that siMIF significantly increased the cell survival inhibition rate in LCC2 cells compared to siNC. The IC_50_ value of 4-OHT was examined after the cells were treated with different concentrations of 4-OHT. The results showed that siMIF significantly reduced the IC_50_ of 4-OHT compared to siNC. ^*∗*^ *P* < 0.05 versus siNC.
